The article "Impact of Tree Cover Loss on Carbon Emission: A Learning-Based Analysis" was published in 2023. Journal: Comput Intell Neurosci.

# Impact of Tree Cover Loss on Carbon Emission: A Learning-Based Analysis

**DOI:** 10.1155/2023/8585839

**Published:** 2023-03-01

**Authors:** Abdul Haleem Butt, Muhammad Ali Jamshed, Ata Ur Rahman, Faiz Alam, Manoj Shakya, Ahmad S. Almadhor, Masoor Ur-Rehman

**Affiliations:** ^1^Department of Creative Technologies, Air University, Islamabad, Pakistan; ^2^James Watt School of Engineering, University of Glasgow, Glasgow, UK; ^3^Department of Computer Science and Engineering, Kathmandu University, Dhulikhel, Nepal; ^4^College of Computer and Information Sciences, Jouf University, Sakakah, Saudi Arabia

## Abstract

Describing the processes leading to deforestation is essential for the development and implementation of the forest policies. In this work, two different learning models were developed in order to identify the best possible model for the assessment of the deforestation causes and trends. We developed autoregressive integrated moving average (ARIMA) model and long short-term memory (LSTM) independently in order to see the trend between tree cover loss and carbon dioxide emission. This study includes the twenty-year data of Pakistan on tree cover loss and carbon emission from the Global Forest Watch (GFW) platform, a known platform to get numerical data. Minimum mean absolute error (MAE) for the prediction of tree cover loss and carbon emission obtained through ARIMA model is 0.89 and 0.95, respectively. The minimum MAE given by LSTM model is 0.33 and 0.43, respectively. There is no such kind of study conducted in order to identify the increase in carbon emission due to tree cover loss most specifically in Pakistan. The results endorsed that one of the main causes of increase in the pollution in the environment in terms of carbon emission is due to tree cover loss.

## 1. Introduction

Global warming is a burning issue causing catastrophic changes and calamities around the world. The increasing occurrence of climate dissipation has been noticed with current global warming that had several biophysical impacts worldwide [1]. One of the main causes of global warming is carbon emission. Sources of carbon emission are both natural and human. Human sources include a variety of man-made actions such as tree logging, forest fires, burning of fossil fuels, cement production, natural gas production, and so on [2, 3].

Hence, the degradation of forests that play an essential role in maintaining a balance in the ecosystem directly adds to global warming. It results in rapid environmental degradation, not only leading to a scarcity of natural resources, decline in quality of life, and long-term public health issues but also inflicting economic losses [4]. Therefore, controlling deforestation can significantly minimize carbon emissions and help improve the environment. Recent studies revealed that the deforestation rate increases with extreme drought and wet years. In another study [5], the authors examined the carbon dioxide emission and climatic effects on major agricultural crop production in Pakistan. The results revealed that the crops such as wheat, maize, sugarcane, cotton, and so on have a constructive association with carbon dioxide emissions. Combating deforestation is being evaluated by cost-effective means of reducing greenhouse gas emissions [6].

The article "Impact of Tree Cover Loss on Carbon Emission: A Learning-Based Analysis" was published in 2023. Journal: Comput Intell Neurosci.

Due to the negative impact of carbon emissions on the environment, there is a lot of ongoing research work to find out the efficient methods that have the ability to predict carbon emissions and determine their causes [7–10]. Learning-based techniques have provided new approaches to prediction problems that represent interactions between variables in a deep and layered hierarchy. ML-based techniques like support vector machines (SVMs) and random forest (RF), as well as DL-based algorithms like recurrent neural network (RNN) and LSTM, have attracted lots of attention in recent years because of their applications in a variety of fields [11–14]. In time series forecasting, DL approaches are capable of identifying data structure and pattern, such as non-linearity and complexity [15, 16]. LSTM has been extensively utilized in time series prediction in [17–21]. Autoregressive integrated moving average (ARIMA) is also another forecasting model [22] that predicts the future values based on the past values. ARIMA is the best model for one-step out-of-sample forecasting and is good for the data which consist of linear and short-term dependency (weekly or hourly) [23].

The rapid advancement in the Internet of Things (IoT) would be a future enhancement of this system. There are multiple privacy-related challenges in IoT architecture during communication that can be addressed using blockchain-enabled IoT architecture [24]. Moreover, there is a need for a decentralized auction-based resource allocation mechanism in edge computing-enabled IoT, which would be helpful to make computer resources closer to the devices [25]. To imporved the data quality during the data communication, few studies foucsed on the age of information (AOI) from the prespective of game theory [26]. Game theory is a useful tool to optimize wireless networks by assisting scarce wireless resource allocation, e.g., bandwidth and channels.

Objective of this study is to develop an accessible methodological approach that allows for rapid evaluation of statistical relationships and trends in forest monitoring data using both ML and DL. In this study, two independent learning models were developed using the autoregressive integrated moving average (ARIMA) model and long short-term memory (LSTM). Moreover, this study also focused on understanding the correlation between tree cover loss and carbon emission by taking Pakistan as a case study. Since, there is no such comprehensive effort found in open literature by the authors, it is a novel attempt in this direction. The remaining part of the paper is arranged as follows. The methodology is discussed in Section 2. In Section 3, results are discussed.  Section 4 describes the conclusion and future work.

The article "Impact of Tree Cover Loss on Carbon Emission: A Learning-Based Analysis" was published in 2023. Journal: Comput Intell Neurosci.

## 2. Methodology

### 2.1. Data Collection

Two time series datasets, i.e., tree cover loss and carbon emission in Pakistan, were taken from the GFW platform [27]. Each dataset consists of past 20 years' information on carbon values added to the environment and the tree cover loss from year 2001 to 2020. It should be noted that a more organized dataset comprising other variables of consideration for this study is not available in the open literature.

Figure 1 shows the proposed methodology of the framework. Following the collection of the dataset, the preprocessing stage is carried out to make the data stationary, as shown in Figure 2. The dataset is then divided into training and testing portions in order to train and evaluate the models. The training component of the dataset is used to train the models, and the testing portion is used for evaluation. The MAP and MAPE error evaluation metrics are evaluated for final analysis of the result.

### 2.2. Data Preprocessing

Figure 2 shows the preprocessing framework. Firstly, we deal with all missing values of the dataset. For any time series forecasting, being stationary is a mandatory property for a statistical model. A series is called stationary if its statistical property does not change with time. To verify this feature in our dataset, we have used the augmented Dickey–Fuller (ADF) test. After applying ADF, it was found that our dataset taken from GFW platform [27] does not fulfill this condition.

In order to make our dataset stationary, we performed a series of transformations such as power log transformation and differencing before applying (ADF) again for the verification. Figure 1 illustrates our adopted methodology in the form of a flowchart. After preprocessing, the dataset is divided into test and training subsets. The training set is used to train the prediction model and the test set is used to evaluate it. The split between the training and test data is kept at 70% and 30%, respectively.

For forecasting, the ARIMA and LSTM models are used to make predictions and are applied on both datasets.

The article "Impact of Tree Cover Loss on Carbon Emission: A Learning-Based Analysis" was published in 2023. Journal: Comput Intell Neurosci.

### 2.3. ARIMA and LSTM Models

The ARIMA model is a generalization of the simpler autoregressive moving average that incorporates the concept of integration. The ARIMA model parameters are as follows:

- p: lag order (previously predicted values).
- d: degree of difference.
- q: order of moving average.

An ARIMA model is a time series forecasting model. It incorporates the properties of two autoregression and moving average models, where in autoregression, lags or previously predicted values are known as “autoregression” while lag or previously predicted error is known as “moving average.” “Difference” is to make time series stationary (also known as integrated stationary time series version).

First step is to determine appropriate hyperparameters of ARIMA, *p*, *h*, and *q*, accurately to predict the behavior of the time series. Then, these hyperparameters are fitted into the training data. Finally, the model fitting residuals are analyzed to check whether the model assumptions are satisfied [6].

This study also utilizes LSTM model, which is a special type of RNN and is able to deal with long-term time dependencies [28]. There are many types of LSTM models that can be used for specific type of time series forecasting problem. In univariate LSTM, single series of observation is required to learn from the past values.

On the contrary, multivariate LSTM makes use of two or more kinds of parallel time series information to learn from the past observations. The basic architecture of univariate LSTM is shown in Figure 3. Basic LSTM network consists of cells that store the data. These cells resemble a transport line that connects one module to another conveying data from the past and gathering the present values [29]. For LSTM, three-layer-based architectures is proposed in this study with a dropout probability of 0.3 and zero non-trainable parameter. The lagged value of time series is used to predict future value with 40,901 learnable parameters.

The LSTM is applied on both of the parameters of carbon emission and tree cover loss with same layers and parameters, and the model for each dataset is trained with 50 epochs. Two separate univariate LSTM models are applied to two different time series variables, i.e., tree cover loss and carbon emission. The models are not only validated based on the difference between observed and predicted values also known as residuals but also exploited for future prediction of tree cover loss association with carbon emission for next three years with upper confidence level of 80% and lower confidence level of 90%.

## 3. Results

### 3.1. Stationary Time Series

Being stationary is an essential condition in time series analysis. Most of the time series models assumed that each point is independent of one another. To check this feature in our time series, ADF is applied. Moreover, to make the time series information stationary, differencing and log transformation are performed. The result of ADF test is shown in Table 1. It can be noted that the value of *P* is less than 0.05. This clearly indicates that after applying log transformation and differencing, we have obtained a stationary time series suitable for further prediction analysis.

The article "Impact of Tree Cover Loss on Carbon Emission: A Learning-Based Analysis" was published in 2023. Journal: Comput Intell Neurosci.

### 3.2. Tree Cover Loss with ARIMA

ARIMA results for tree cover loss are shown in Figures 4 and 5. The model is trained with multiple order of ARIMA. The minimum MAE for tree cover loss is 0.95 with ARIMA (1, 1, 1). Similarly, the minimum MAE for tree cover loss is 1.4 and 1.2 with ARIMA (1, 2, 1). Values of *p*, *d*, and *q* are cross-checked using auto ARIMA function in Python.  Figure 4 depicts the train (actual) and test (predicted) data showing that the data predict some trends and are at a right scale. In Figure 5, data for past twenty years (2001–2020) are utilized to train the model for prediction of tree cover loss for next five years. The results indicate an increase in tree cover loss in the coming years.

### 3.3. Carbon Emission with ARIMA

Figures 6 and 7 show the carbon emission results using ARIMA. The model is trained with multiple order of ARIMA. The minimum MAE of 1.20 and mean absolute percentage error (MAPE) of 1.24 are obtained for carbon emission forecasting with ARIMA order of (1, 1, 1) and (1, 2, 1), respectively. The twenty-year data, from 2001 to 2020, are used for the model training. The same model is further exploited to carry out forecasting carbon emission over next five years. The results indicate an increase in the carbon emission for this coming period.

The two results also exhibit that increase in the carbon emission has significant and similarly directed impact on the tree cover loss.

### 3.4. Tree Cover Loss with LSTM

LSTM has also been applied on the same dataset to compare the results with ARIMA model for tree cover loss. Figures 8 and 9 demonstrate the results for this study. Training and testing loss decay per epoch is shown in Figure 8 while Figure 9 illustrates the tree cover loss prediction for next three years, i.e., 2023–2025.

### 3.5. Carbon Emission with LSTM

Figures 10 and 11 show the results of LSTM-based carbon emission. The LSTM model is trained up to 50 epochs for both tree cover loss and carbon emission. It is observed from Figure 10 that the train and testing loss is decreasing over time after each epoch while using LSTM. The results indicate that a linear correlation exists between the carbon emission and tree cover loss. Future predictions of the LSTM model also reflect an increasing pattern of the carbon emission.

The article "Impact of Tree Cover Loss on Carbon Emission: A Learning-Based Analysis" was published in 2023. Journal: Comput Intell Neurosci.

### 3.6. Comparison of ARIMA and LSTM

The ARIMA model works by filtering high-frequency noise from data, detecting local patterns based on linear dependencies, and predicting future trends [30]. In addition, the ARIMA model converts tree cover losses and carbon emission features into special temporary variables before matching them and only considers the linear portion of the series [31]. The ARIMA model is simple and forthright and only requires to adjust the values of *p*, *d*, and *q*. The ARIMA model, however, is unable to deal with the non-linear relationship between the tree cover loss and carbon emissions.

On the contrary, the neural network such as LSTM can deal with both linear and non-linear patterns [32]. LSTM is a type of RNN that is meant to learn temporal patterns, capture non-linear dependencies, and preserve relevant memory for a longer period of time, resulting in achieving more accurate predictions [33].

Working of the two approaches, ARIMA and LSTM, for tree cover loss and carbon emission prediction is investigated using mean average precision (MAP) and MAPE evaluation matrices. Results are summarized in Table 2. It is observed that MAP obtained through LSTM is 0.33 while MAPE is 0.25. For carbon emission, LSTM gives MAP of 0.43 and MAPE of 0.40.

The results clearly show that LSTM has performed better than the ARIMA model in estimating and predicting tree cover loss and carbon emission for the analyzed data, hence ratifying that LSTM architecture is more suitable for time series prediction than ARIMA. The results also reflect the strong reliance and linear relationship between the tree cover loss and carbon emission.

## 4. Conclusion

In this work, a detailed analysis of tree cover loss and carbon emission data is carried out using ARIMA and LSTM techniques. 20-year data, from 2001 to 2020, are utilized to train and test the models and get predictions for next 5 years. The relationship between the two environmental factors is also established. The results have shown that temporal variations in the trend component of both carbon emission and tree loss cover are remarkably associated with each other. It has established that increase in the tree cover loss directly affects carbon emission in the atmosphere. Carbon emission could be one of the significant causes of the tree cover loss and deforestation.

Working of LSTM is found to be more vigorous in these prediction studies. Though very significant, this study is limited by the limited data availability. Both ARIMA and LSTM models showed the same trends. However, LSTM is a model that can learn the long-term dependencies, and it can remember the information that is processed in the model for a very long time [22]. In terms of computational time, the ARIMA models consume more time when using the rolling forecast method, and it is unfeasible to train new models when the orders of *p*, *d*, and *q* increase [34]. LTSM models take significantly less time to train, and once trained, constant predictions can be obtained, while ARIMA models need to be retrained.

The article "Impact of Tree Cover Loss on Carbon Emission: A Learning-Based Analysis" was published in 2023. Journal: Comput Intell Neurosci.

Future aspects of this study include better understanding of carbon emission impact and control by considering more factors such as wood fuel, fire, and timber harvest. Inclusion of more factors and parameters can improve the overall prediction accuracy of the models while providing a broader understanding of causes of carbon emission. If more variables that contribute to carbon emissions and deforestation are taken into account, the work described in this paper will be more sophisticated.

## Figures and Tables

**Figure 1:** Hierarchical representation of the proposed methodology used to carry out forecasting.

**Figure 2:** Hierarchical illustration of data preprocessing framework.

**Figure 3:** Architecture of basic LSTM network for univariate prediction.

**Figure 4:** Actual versus predicted tree cover loss using ARIMA model.

**Figure 5:** Train versus future predicted tree cover loss using ARIMA model.

**Figure 6:** Actual versus predicted carbon emission using ARIMA model.

**Figure 7:** Actual versus predicted carbon emission using ARIMA model.

**Figure 8:** Loss decay per epoch for tree cover loss using LSTM.

**Figure 9:** Actual versus predicted tree cover loss using LSTM.

**Figure 10:** Loss decay per epoch for carbon emission using LSTM.

**Figure 11:** Actual versus predicted carbon emission using LSTM.

**Table 1:** ADF test results.

Tree cover loss		Carbon emission	

Test statistic	−4.1812	Test statistic	−3.7851
*P* value	0.00078	*P* value	0.00532
Lag used	0.00000	Lag used	0.00000
No. of abbreviations used	18.0000	No. of abbreviations used	15.0000
Critical value (1%)	−3.8590	Critical value (1%)	−2.0521
Critical value (5%)	−3.0420	Critical value (5%)	−2.6710
Critical value (10%)	−2.6609	Critical value (10%)	−1.7219

**Table 2:** Comparison of ARIMA and LSTM for tree cover loss and carbon emission prediction.

Tree cover loss			Carbon emission	
Models	MAP	MAPE	MAP	MAPE
ARIMA (1, 2, 1)	1.34	4.45	1.24	1.20
ARIMA (1, 1, 1)	0.95	4.35	0.89	5.65
ARIMA (1, 2, 2)	3.81	9.10	3.58	8.21
LSTM	0.33	0.25	0.43	0.40

## Data Availability

The data used to support the findings of this study are available publicly on Global Forest Watch.
